# LRG1 modulates epithelial-mesenchymal transition and angiogenesis in colorectal cancer via HIF-1α activation

**DOI:** 10.1186/s13046-016-0306-2

**Published:** 2016-02-09

**Authors:** Jingjing Zhang, Lingyin Zhu, Jingyuan Fang, Zhizheng Ge, Xiaobo Li

**Affiliations:** State Key Laboratory for Oncogenes and Related Genes, Key Laboratory of Gastroenterology & Hepatology, Ministry of Health, Division of Gastroenterology and Hepatology, Ren Ji Hospital, School of Medicine, Shanghai Jiao Tong University, Shanghai Cancer Institute, Shanghai Institute of Digestive Disease, 145 Middle Shandong Road, Shanghai, 200001 China

**Keywords:** LRG1, HIF-1α, EMT, Angiogenesis, Colorectal cancer

## Abstract

**Background:**

Leucine-rich-alpha-2-glycoprotein 1 (LRG1) has been reported to be involved in several tumors, whether it participates in colorectal cancer (CRC) progression remains unclear. Here, we investigated the biological function and underlying molecular mechanisms of LRG1 in CRC.

**Methods:**

The mRNA and protein levels of LRG1 were assessed in CRC tissues through RT-PCR and immunohistochemistry, respectively. HCT116 and SW480 cells were treated with LRG1 siRNA, control siRNA, or recombinant LRG1. Transwell invasion assays and wound healing assays were performed to evaluate the invasion and migration of CRC cells. Epithelial-to-mesenchymal transition (EMT) markers of E-cadherin, VDR, N-cadherin, α-SMA, Vimentin and Twist1 were detected by RT-PCR and western blot. Enzyme-linked immunosorbent assay was used to measure the secretion level of VEGF-A. Conditioned medium from CRC cells was collected for endothelial cell migration, tube formation and aortic ring sprouting assays.

**Results:**

LRG1 was overexpressed in CRC tissues and associated with cancer aggressiveness. LRG1 was further found to induce the EMT process, as well as CRC cell migration and invasion capacity. In addition, LRG1 promoted VEGF-A expression in CRC cells and contributed to tumor angiogenesis. Furthermore, HIF-1α could be induced by LRG1 in a concentration- and time-dependent manner, which was responsible for LRG1-induced VEGF-A expression and EMT.

**Conclusions:**

The present study suggests that LRG1 plays a crucial role in the progression of CRC by regulating HIF-1α expression, thereby may be a promising therapeutic target of CRC.

## Background

Despite advances in early diagnosis and comprehensive therapy, colorectal cancer (CRC) remains one of the leading causes of cancer death worldwide. The prognoses of CRC patients were often poor due to recurrence and metastasis, especially for those diagnosed at advanced stages. The 5-year survival rate is only 12 % for CRC patients with distant metastasis [1]. Hence, elucidating the molecular events involved in CRC and identifying novel biomarker and therapeutic targets is indispensible and urgent for the clinical outcome of CRC.

Leucine-rich-alpha-2-glycoprotein1 (LRG1) is the founding member of leucine-rich repeat (LRR) family, which was first isolated from human serum in 1977 [2]. It is a secreted glycoprotein and contains eight repeating consensus sequences, each of which consists of 24 amino acid residues [3]. LRG1 has been reported to be involved in immune response, cell proliferation, cell migration, cell apoptosis and neovascularization [4–7]. LRG1 is overexpressed in several types of carcinomas, including pancreatic, bladder, ovarian, and biliary tract cancer [8–11]. LRG1 was shown to bind to the transforming growth factor-beta (TGF-β) accessory receptor and modulate Smad1/5/8 signalling pathway, resulting in promotion of angiogenesis in endothelial cells [7]. It was reported that LRG1 was a target of miR-335 and contribute to the migratory and invasive ability of neuroblastoma cell [5]. However, little is known about the biological function of LRG1 in colorectal cancer.

To reveal the signaling proteins downstream of LRG1, we performed a gene microarray and found that several key proteins involved in epithelial-to-mesenchymal transition (EMT) were affected by depletion of LRG1 in CRC cells. EMT is a pathological process that epithelial cells lose their characteristic of cell polarity and adhesion, while acquire a mesenchymal phenotype [12]. EMT process results in enhanced ability of mobility and invasiveness for carcinoma cells, which is considered as a crucial early step in cancer progression and metastasis [13–15]. Besides, hypoxia-inducible factor-1α (HIF-1α) and vascular endothecial growth factor A (VEGF-A) was significantly downregulated in LRG1-knockdown CRC cells. HIF-1α is the oxygen-regulated subunit of HIF-1, which is the most important transcriptional regulator in response to hypoxia. HIF-1α participates in the key steps in carcinogenesis such as cell survival, angiogenesis and metastasis, through transcriptional activation of targeted genes [16, 17]. Notably, HIF1α has been identified as an important mediator of EMT in tumor cells via activation of Twist, Snail, and SIP1 [18, 19]. The mechanisms underlying HIF-1α-induced EMT in CRC have not been completely determined. Therefore, LRG1 might be associated with the EMT and angiogenesis in CRC.

In the present study, we investigated the expression level of LRG1 in CRC tissues and explored the role of LRG1 in CRC cell invasion, EMT, and endothelial cell activities. We also aimed to validate the promotion effect of LRG1 on HIF-1α expression and test the hypothesis that HIF-1α is involved in LRG1-induced EMT and angiogenesis in CRC.

## Methods

### Cell culture and LRG1 treatment

Human colorectal carcinoma cell lines, SW480 and HCT116, were cultured in RPMI 1640 medium supplemented with 10 % fetal bovine serum (FBS) in humidified 5.0 % CO_2_ atmosphere at 37 °C. Human umbilical vein endothelial cells (HUVEC) were maintained in DMEM containing 10 % FBS. Recombinant LRG1 was purchased from R&D Systems and added into the culture medium at concentration of 50–1000 ng/ml for indicated time before harvesting.

### Small interfering RNA silencing

Transfection of siRNA was performed using Lipofectamine 2000 (Invitrogen, USA) according to the manufacturer’s protocol. The transfection reagent was replaced by complete medium after incubation for 6 h, and cells were harvested 24 h or 48 h later. The siRNA oligos for LRG1 (#1: sense, 5′-CCUCUAAGCUCCAAGAAUUTT-3′ and antisense, 5′-AAUUCUUGGAGCUUAGAGGTT-3′; #2: sense, 5′-GCAAUUAGAACGGCUACAUT T-3′ and antisense, 5′-AUGUAGCCGUUCUAAUUGCTT-3′), HIF-1ɑ (#1: sense, 5′-GGAA AGAGACUCAUAGAAA-3′ and antisense, 5′-UUUCUAUGACUCUCUUUCC-3′; #2: sense, 5′-GCACAGGCCACATTCACGTATAT-3′ and antisense, 5′- GGTTCACAAATCAGC ACCAAGC-3′), and a non-targeting control siRNA were purchased from GenePharma (China).

### RNA extraction and quantitative real-time PCR

Total RNA was extracted by Trizol (Invitrogen, USA), and cDNA was synthesized using the PrimeScript TM RT Reagent Kit (Perfect Real Time, TaKaRa, Japan). Quantitative real-time PCR was performed in a 10ul total volume containing SYBR Green (SYBR® Premix Ex Taq TM II, TaKaRa, Japan) on an Applied Biosystems 7900 quantitative PCR system. The primers used were as follows: LRG1, 5′-GTTGGAGACCTTGCCACCT-3′ and 5′-GCTTGTTGCCGTTCAGGA-3′; HIF-1*α*, 5′-TGCTAATGCCACCACTACC-3′ and 5′-TG ACTCCTTTTCCTGCTCTG-3′; VEGF-A, 5′-CTTTCTGCTGTCTTGGGTG-3′ and 5′-ACT TCGTGATGATTCTGCC-3′; Twist1, 5′-AGTCCGCAGTCTTACGAGGA-3′ and 5′-GCCAG CTTGAGGGTCTGAAT-3′; E-cadherin, 5′-TACACTGCCCAGGAGCCAGA-3′ and 5′-TGG CACCAGTGTCCGGATTA-3′; N-cadherin, 5′-TTTGATGGAGGTCTCCTAACACC-3′ and 5′-ACGTTTAACACGTTGGAAATGTG-3′; VDR, 5′-GATGCCCACCACAAGACCTA-3′ and 5′-CGGTTCCATCATGTCCAGTG-3′; Vimentin, 5′-TGAGTACCGGAGACAGGTGCA G-3′ and 5′-TAGCAGCTTCAACGGCAAAGTTC-3′; α-SMA, 5′-CGTGGCTACTCCTTCGT G-3′ and 5′-TGATGACCTGCCCGTCT-3′; β-actin, 5′-TGGCACCCAGCACAATGAA-3′ and 5′-CTAAGTCATAGTCCGCCTAGAAGCA-3′. Relative expression of each specific gene was determined in accordance with the 2^−ΔΔCt^ method, using β-actin as the internal standard. Each experiment was performed as triplicate, and data was presented as mean ± SEM.

### Clinical specimens and immunohistochemistry

Human CRC tissues and adjacent non-cancerous tissues were obtained from patients who underwent surgical resection at Renji Hospital. Histological diagnoses were performed by expert pathologists. The study was approved by the Ethics Committee of Renji hospital, and written informed consent was obtained from all patients included in this study.

Paraffin-embedded specimens of 68 colorectal cancers and 32 normal colorectal tissues were selected for immunohistochemistry. Briefly, antigen retrieval was performed with 10 mM citrate buffer (Ph 6.0) using microwave. Sections were incubated with anti-LRG1 antibody (1:100, Abcam, USA) overnight at 4 °C, followed by HRP-conjugated secondary antibody. LRG1 expression was quantified based on the intensity of staining (scored as: 0, no staining; 1, weak staining; 2, moderate staining; 3, strong staining) and the percentage of positive tumor cells (scored as: 0, less than 5 %; 1, 5–25 %; 2, 26–50 %; 3, > 51 %). The final score was calculated as the product of two parameters, and at least 3 points was considered as positive.

### Invasion and migration assay in vitro

The cell invasion assay was carried out using chambers with filters (pore size of 8-um), coated with Matrigel. The cells (2*10^5^ cells per well) were seeded into the upper chamber in serum-free medium, while medium with 20 % FBS was applied to the lower chamber. For endothelial cells, conditioned medium was added to the lower chamber. After incubation for 48 h, invasive cells on the bottom surface of the membrane were fixed with 4 % formaldehyde, stained with crystal violet, and counted in five random microscopic fields for each replicate (original magnification, 200×).

The migration ability of cells was measured through wound healing assay. Cells were cultured in 6-well plates to reach 90 % confluence. The cell monolayers were scraped with a 100-ul pipette tip, washed twice with PBS, and cultured in serum-free medium. After 24 h and 48 h, the scratch area was photographed (original magnification, 200×).

### Conditioned medium and enzyme-linked immunosorbent assay

CRC cells cultured in 6-well plates were treated with LRG1 for 24 h. Thereafter, cells were washed three times and changed to fresh serum-free medium for additional 24 h. The supernatants were harvested, centrifuged at 3500 rpm for 5 min, and stored at−80 °C until used as conditioned medium (CM). Tumor-derived VEGF-A in the medium was quantified by enzyme-linked immunosorbent assay (ELISA). VEGF-A concentration was determined using ELISA Kit (R&D Systerms Europe, UK) according to the manufacturer’s instructions.

### Endothelial cell tube formation assay

Matrigel (BD Biosciences, CA) was laid into a 48-well plate and polymerized at 37 °C for 30 min. Then, 3 × 10^4^ HUVECs were seeded into each well of pre-coated 48-well plate and incubated with conditioned medium. After 8 h, capillary-like tubes were photographed (original magnification, 100×) from four randomly chosen fields, and the total number of complete tubular structures was quantified.

### Aortic ring sprouting assay

Aortas were excised from 8-week-old Sprague–Dawley rats and dissected into rings of 1 mm. Aortic rings were embedded in Matrigel (BD Biosciences, California, USA) in a 48-well culture plate. CM was added to the wells in a final volume of 200ul culture medium. The aortic rings were incubated at 37 °C for 6 days with medium replaced every other day. On day 6, the microvessel sprouting was photographed and scored from 0 (least positive) to 5 (most positive) in a double-blinded manner as previously described [20]. Three independent experiments were carried out with five rings per group in each assay. Representative micrographs were shown.

### Western blot

Whole-cell protein extracts were prepared with RIPA buffer containing a protease inhibitor mixture. Protein concentrations were determined using BCA Protein Assay. Equal amounts of total protein were separated by SDS–polyacrylamide gel electrophoresis, transferred onto the polyvinylidene difluoride membrane, and blocked with 5 % fat-free milk. The membranes were incubated with primary antibodies overnight at 4 °C, followed by HRP-conjugated secondary antibodies for 1 h at room temperature. The immune complexs were detected using a chemiluminescence kit (SuperSignal ECL Kit, Thermo Fisher, USA). Antibody for LRG1 was purchased from Abcam (USA), and other antibodies were all purchased from Cell Signaling Technology Inc (USA). Intensity of the protein bands was quantified by Image J software and normalized to that of β-actin.

### Statistical analysis

Statistical analysis was carried out using SPSS 20.0 software (SPSS, Chicago, IL, USA). Quantitative data were expressed as the means ± SEM, and comparisons between every two groups were performed with Student *t* test or paired *t* test. The association between LRG1 staining and the clinicopathologic features of CRC patients were examined by Chi-square tests. *P*-value <0.05 was considered statistically significant.

## Results

### LRG1 expression was increased in human CRCs and correlated with tumor progression

To investigate the mRNA expression level of LRG1 in CRC, we analysed the microarray data from two Oncomine Cancer Microarray databases (GSE20916 and GSE20842) and revealed remarkable overexpression of LRG1 in CRC tissues than normal tissues (Fig. 1a). Next, we performed real-time RT-PCR to assess LRG1 expression in 30 cases of CRC tissues and matched normal tissues. Similar result was observed that LRG1 was significantly overexpressed in CRC tissues, compared with corresponding normal tissues (*P* < 0.0001, Fig. 1b). Immunohistochemistry was performed to examine LRG1 protein in 68 CRC and 32 normal paraffin-embedded tissues. Positive staining of LRG1 was mainly distributed in the cytoplasm and cytomembrane of CRC cells (Fig. 1c). Positive expression rate of LRG1 was 66.18 % (45/68) in CRC tissues, significantly higher than that of normal colorectal mucosa (31.25 %, 12/32) (*P* = 0.007). The clinicopathologic features of the 68 CRCs were summarized in Table 1. LRG1 expression was significantly correlated with deeper invasion depth (*P* = 0.032) and lymph node metastasis (*P* = 0.013). There was no significant correlation between LRG1 expression and other clinicopathological characteristics, including age, gender, location, tumor size and distal metastasis.

**Fig. 1:** LRG1 was overexpressed in CRC tissues. **a** Overexpression of LRG1 mRNA in CRC tissues than normal tissues based on the microarray data from GSE20916 and GSE20842. **b** RT-PCR analysis of LRG1 mRNA expression in 30 pairs of CRC and adjacent non-tumor tissues. The expression levels of LRG1 were normalized to those of β-actin (*P* < 0.0001, paired t test). **c** Representative immunohistochemical staining of LRG1 in human samples of normal tissue, early CRC tissue, and advanced CRC tissue (Original magnification: ×200 and 400×). *Scale bar* represents 50 μm

**Table 1:** Correlation between LRG1 expression and clinicopathological parameters of CRCs

	n	LRG1 expression		*P* values
		Negative	Positive	
Age				
< 60	37	12	25	0.791
≥ 60	31	11	20	
Gender				
Male	41	13	28	0.649
Female	27	10	17	
Location				
Right colon	21	9	12	0.396
Left colon	18	4	14	
Rectum	29	10	19	
Tumor diameter				
< 5 cm	35	11	24	0.667
≥ 5 cm	33	12	21	
T stage				
T1 + T2	32	15	17	0.032
T3 + T4	36	8	28	
Lymph nodes metastasis				
Negative	39	18	21	0.013
Positive	29	5	24	
Distant metastasis				
Negative	63	23	40	0.242
Positive	5	0	5	

### LRG1 influenced CRC cell migration, invasion and EMT

The overexpression of LRG1 in CRCs suggested that LRG1 might play a role in its migration and invasion capability. To investigate the function of LRG1 in CRC cells, we knocked down LRG1 by transfection of specific siRNA. Both mRNA and protein levels of LRG1 were efficiently depleted in HCT116 and SW480 cells (Fig. 2a). Transwell and wound healing assay were used to examine invasion and migration of CRC cells. In transwell assays, knockdown of LRG1 significantly reduced the number of cells invaded through the membrane compared with the control (Fig. 2b). Likewise, wound closure ratio was markedly reduced to 48 and 61 % respectively (*P* both <0.05) in LRG1-siRNA transfected HCT116 and SW480 cells (Fig. 2c). Next, we examined the expression of EMT markers following knockdown of LRG1. Real-time RT-PCR and western blot analysis showed that epithelial biomarkers of E-cadherin and VDR were increased in LRG1-depleted CRC cells, whereas mesenchymal biomarkers of N-cadherin, α-SMA and Vimentin were decreased. Furthermore, we investigated whether the EMT-related transcription factors were involved in LRG1-promoted EMT. Results showed that Twist1 expression was significantly decreased by LRG1 knockdown in both cell lines (Fig. 3a and b). These results suggested that LRG1 can enhance CRC cell invasion and induce EMT.

**Fig. 2:** Knockdown of LRG1 repressed the invasion capacity of CRC cells. **a** RT-PCR and Western blot analyses showed effective downregulation of LRG1 following siRNA transfection. **b** HCT116 and SW480 cells transfected with LRG1 siRNA or control siRNA were seeded in the upper chamber. After 48 h, the cells invaded through the membrane were stained and counted in five random microscopic fields (200×). **c** LRG1- and control-siRNA transfected HCT116 and SW480 cells were wounded with pipette and wound closure percentage was quantified 48 h after scratch relative to that at 0 h. *P < 0.05 compared to the control cells. *Scale bar* represents 100 μm

**Fig. 3:** Knockdown of LRG1 prevents the mesenchymal transition. **a** and **b** Expression of EMT-associated markers in CRC cells with LRG1 siRNA or control siRNA were measured by RT-PCR and western blot assays. *P < 0.05 compared to the control cells

### LRG1 supplementation enhanced expression and secretion of VEGF-A and promotes endothelial cells migration and tube formation

Angiogenesis is an essential step in tumor metastasis. Given that LRG1 was reported to be a new regulator of angiogenesis, we determined whether LRG1 was involved in CRC angiogenesis. Our data implied that treatment with human rLRG1 for 24 h concentration- dependently increased VEGF-A mRNA expression and protein secretion level in both SW480 and HCT116 cells (Fig. 4a). Similarly, VEGF-A expression was elevated by stimulation with rLRG1 in a time-dependent manner (Fig. 4b). To further investigate the role of LRG1 in angiogenesis, we collected the CM derived from HCT116 cells incubated in the presence or absence of rLRG1 (500 ng/ml). The CM was then applied to HUVECs for transwell migration, tube formation and aortic ring sprouting assays. As shown in Fig. 4c, CM from CRC cells exposed to LRG1 promoted endothelial cell migration. In tube formation assays, the cumulative number of tubular structures formed by HUVECs in CM from LRG1-treated CRC cells was significantly increased (2.6 fold, Fig. 4d). Microvessel sprouting from aortic rings was significantly stimulated in the presence of CM from LRG1-treated CRC cells (Fig. 4e). In these assays, the promotion effect of LRG1 on endothelial cell behaviors was blocked by LRG1 mAb. These results provided evidence for the role of LRG1 in promotion of angiogenic capability in colorectal carcinomas.

**Fig. 4:** LRG1 promoted VEGF-A expression and angiogenesis. **a** HCT116 and SW480 cells were stimulated with rLRG1 (0–1000 ng/ml) for 24 h, and VEGF-A expression was quantified by RT-PCR and ELISA. **b** CRC cells were stimulated with rLRG1 (500 ng/ml) for indicated hours, and VEGF-A expression was quantified by RT-PCR and ELISA. **c** and **d** The medium of HCT116 cells incubated in the presence or absence of LRG1 (500 ng/ml) and LRG1 antibody (10 μg/ml) was collected and then applied to HUVECs for transwell migration assay and tube formation assay. **e** Effect of CM from LRG1-induced HCT116 cells on the aortic ring sprouting assay. Representative photos were shown and data were summarized from 3 independent experiments. *Compared to the control group, *P* < 0.05. *Scale bar* represents 100 μm

### HIF-1α was essential for LRG1-mediated EMT and angiogenesis

HIF-1α was a critical regulator in both tumor angiogenesis and hypoxia-induced EMT. To examine whether LRG1 would enhance HIF-1α expression, CRC cells were treated with rLRG1 for 24 h. HIF-1α mRNA expression was induced at 100 ng/ml and reached the maximum level at 1000 ng/ml (Fig. 5a). Protein expression of HIF-1α was also increased following stimulation with rLRG1 in a concentration-dependent manner in SW480 cells. LRG1 stimulation also resulted in increased expression of VEGF-A, Twist1 and N-cadherin, while decreased E-cadherin expression (Fig. 5b). Further we determined the role of HIF-1α in LRG1-induced VEGF-A overexpression and EMT. Transfection with siRNA successfully silenced the mRNA and protein levels of HIF-1α expression in SW480 cells (Fig. 5c). Secretion of VEGF-A by SW480 cells was elevated in the presence of LRG1, and the effect was abolished by knockdown of HIF-1α (Fig. 5d). Knockdown of HIF-1α also reversed LRG1-induced EMT phenotype, increasing E-cadherin expression, and decreasing Twist1 and N-cadherin expression (Fig. 5e). As shown in Fig. 5f, silencing HIF-1α inhibited the enhanced invasion ability of CRC cells induced by LRG1. These results strongly implied that HIF-1α is implicated in LRG1-induced CRC cells invasiveness, EMT and angiogenesis.

**Fig. 5:** The role of HIF-1α in LRG1-induced EMT and VEGF-A expression. **a** HIF-1α mRNA expression in HCT116 and SW480 cells stimulated with indicated concentrations of LRG1 for 24 h was measured by RT-PCR. β-actin was used as the internal control. **b** The protein levels of HIF-1α, Twist1, E-cadherin, and N-cadherin in response to LRG1 in SW480 cells were measured by western blot. **c** HIF-1α expression was knocked down in siRNA-transfected SW480 cells at both mRNA and protein levels. **d** SW480 cells were transfected with HIF-1α or control siRNA for 24 h, and treated with or without rLRG1 (500 ng/ml) for additional 24 h. Secretion of VEGF-A from SW480 cells was quantified by ELISA. **e** HIF-1α, VEGF-A, E-cadherin, N-cadherin and Twist1 expressions were detected by western blot. **f** SW480 cells were harvested and applied for transwell invasion assays. The numbers of invasive cells (five random fields) were expressed as means ± SEM of three independent experiments. *Compared to the control group, *P* < 0.05. *Scale bar* represents 100 μm

## Discussion

It was reported that plasma levels of LRG1 in patients with CRC were higher than those with adenomatous polyps, which might be a novel biomarker for the progression from colorectal adenoma to carcinoma [21]. In our study, we demonstrated that LRG1 expression was significantly increased in CRC tissues compared with normal tissues. In addition, expression level of LRG1 was positively associated with deeper invasion depth and lymphatic metastasis. These results imply that LRG1 may be involved in colorectal cancer initiation and progression, which is in agreement with published studies of ovarian cancer and biliary tract cancer [10, 11]. However, LRG1 has been reported to act as a tumor suppressor in hepatocellular carcinoma and endometrial carcinoma [22, 23]. The discrepancy of LRG1 function in certain kinds of cancers may be due to its tissue specificity.

Although LRG1 is found to be implicated in various kinds of malignant carcinomas and benign diseases, the biological functions of LRG1 have not been fully elucidated. LRG1 has been predicted to play a role in cell adhesion and cell migration due to its leucine-rich repeats and tendency to bind extracellular matrix proteins [24]. A recent study showed that LRG1 promoted proliferation, migration and invasion of glioma cells, as well as downregulated the expression of E-cadherin [25]. Our experiments demonstrated that knockdown of LRG1 by siRNA significantly attenuated the migratory and invasive potency of CRC cells. Moreover, depletion of LRG1 caused a shift from mesenchymal markers to epithelial markers, which was upregulation of E-cadherin and VDR, and downregulation of N-cadherin, α-SMA and Vimentin. Meanwhile, stimulation with recombinant LRG1 induced EMT and enhanced cell invasion. The expression of Twist1, a well known EMT-promoting transcriptional factor, was also found to be positively regulated by LRG1. Our findings identified LRG1 as a novel inducer of EMT and a potential enhancer of the metastatic potential in colorectal cancer.

Sustained angiogenesis is known as an essential part in the unrestrained growth of tumors and metastasis of cancer cells to distant organs. It has been reported that LRG1 influences endothelial cells proliferation, migration, tube formation, and promotes blood vessel growth in *ex vivo* models of angiogenesis [7]. Whether LRG1 could regulate angiogenesis and be a promising anti-angiogenic therapy target in colorectal cancer were unknown. Our study revealed that treatment of CRC cells with rLRG1 induced the expression of critical pro-angiogenic molecules including HIF-1α and VEGF-A. Cytokines derived from the tumor microenvironment could facilitate the activities of endothelial cells and promote angiogenesis [26, 27]. Therefore, we used the conditional medium from CRC cells to determine whether LRG1 expression modulated endothelial cell migration and tube formation, both of which are critical indicators of angiogenic ability. We found that endothelial cell cultured with CM from rLRG1-stimulated CRC cells exhibited an increased migration and tube formation capacity. Taken together, our results indicated that overexpression of LRG1 in CRC cells might promote the secretion of pro-angiogenic factors like VEGF-A, thus contributing to CRC angiogenesis. Further studies with *in vivo* experiments are needed to demonstrate the biological role of LRG1 in CRC angiogenesis and metastasis.

In this study, we found that treatment of CRC cells with LRG1 promoted the mRNA and protein expression of HIF-1α. Hypoxia or overexpression of HIF-1α is associated with resistance to cancer chemotherapy and increased patient mortality [28]. HIF-1α was reported to be overexpressed in CRC and correlated with poor prognosis [29, 30]. Since the critical role of HIF-1α in tumor progression and metastasis, inhibition of HIF-1α was considered as a promising therapeutic strategy. HIF-1α, the regulatory subunit of HIF-1, is mainly regulated in an oxygen-dependent manner. HIF-1α is rapidly degraded under normoxic conditions through various post-translational modifications of hydroxylation, ubiquitination and ultimate proteasomal degradation [31]. However, several stimuli such as EGF, TGF-β, and IGF-1 can induce HIF-1α accumulation under normoxia, at various levels of transcription, translation, and protein stability in a cell-type-specific manner [32–34]. Consistent with the role of HIF-1α in inducing EMT and metastatic phenotypes, our results indicated HIF-1α to be involved in LRG1-induced EMT, since knockdown of HIF-1α blocked the mesenchymal phenotype and invasive capacity induced by LRG1. Moreover, HIF-1α knockdown abrogated the LRG1-induced VEGF-A expression, which acts as a key downstream target of HIF-1α. These data suggested that LRG1 may target the HIF-1α pathway to induce CRC cell invasion and angiogenesis. A recent study showed that LRG1 overexpression activated the canonical TGF-β signaling pathway and enhanced the invasiveness of glioma cells, which could be reversed by TGF-β signaling pathway inhibitor [24]. It has been shown that TGF-β stimulates HIF-1α accumulation and that HIF-1α mediates TGF-β-induced EMT [35]. It is not clear whether LRG1 activates the transcription of HIF-1α directly or via TGF-β pathway.

## Conclusion

In summary, this is a preliminary study to investigate the role of LRG1 in colorectal cancer. Our results provided evidence for LRG1 function as a novel inducer of EMT and angiogenesis in colorectal cancer, which was at least partially through promotion of HIF-1α expression. Thus, LRG1 may be a potential biomarker and therapeutic target for colorectal cancer. Further researches are still needed to clarify the molecular mechanisms and therapeutic benefits of LRG1 on CRC and other malignancies.

## Abbreviations

LRG1: leucine-rich-alpha-2-glycoprotein 1
CRC: colorectal cancer
EMT: epithelial-to- mesenchymal transition
HIF-1α: hypoxia-inducible factor-1α
VEGF-A: vascular endothecial growth factor A
